The article "Correlation Analysis of Positive Therapy Based on High Content Image Analysis Technology on Posttraumatic Nerve Growth in Patients with COVID-19 in the Context of Intelligent Medical Treatment" was published in 2022. Journal: Contrast Media Mol Imaging.

# Correlation Analysis of Positive Therapy Based on High Content Image Analysis Technology on Posttraumatic Nerve Growth in Patients with COVID-19 in the Context of Intelligent Medical Treatment

**DOI:** 10.1155/2022/9165764

**Published:** 2022-07-19

**Authors:** Ting Zheng, Jie Lin, Liwen Tu, Jiaying Hu, Weiping Wei

**Affiliations:** Department of Emergency, Shanghai Jiaotong University Affiliated Sixth People's Hospital, Shanghai, China

## Abstract

**Objective:**

To investigate the correlation between posttraumatic stress disorder (PTSD) and the incidence of anxiety, depression, and mental disorders in patients with novel coronavirus pneumonia.

**Methods:**

Novel coronavirus pneumonia patients in Wuhan from 2020 to April were selected for treatment from hospitals and isolation wards from 1 to April. 70 rehabilitated patients were randomly divided into the control group (35 patients) and the observation group (35 patients) who were treated with conventional therapy. Positive therapy and full perfusion therapy were introduced on the basis of conventional therapy, and the related performances of different patients were observed and evaluated.

**Results:**

The anxiety, depression, and incidence rate of related psychotic patients in the observation group after treatment were significantly reduced. Patients could maintain a good mood, increase their confidence in conquering diseases, and promote their early recovery.

**Conclusion:**

Active treatment of novel coronavirus pneumonia has positive effects on posttraumatic growth of new crown pneumonia patients, relieving anxiety and negative emotions, improving emotional control, eliminating bad emotions, actively guiding patients, and promoting psychological rehabilitation of patients.

## 1. Introduction

The novel coronavirus pneumonia (coronavirus disease 2019, COVID-19), referred to as “new crown pneumonia,” refers to pneumonia caused by 2019 new coronavirus infection. The WHO named it as “2019 coronavirus” disease (Virus). A novel coronavirus pneumonia outbreak caused by new coronavirus SARS-CoV-2 in Wuhan, China, is a common disease that spreads through the virus. The new transmission routes mainly include direct transmission (clothes and body contact), aerosol transmission (the patient's droplets are discharged into the air, and the water will form aerosols after evaporation), droplet transmission (the body is discharged through speaking, coughing, sneezing, etc.), and other transmission modes. The transmission speed is very fast, and the transmission range is very wide [1]. Up to now (May 9, 2020), it has caused 84416 confirmed cases and 4643 deaths in China. This large-scale public health incident has seriously affected the development of China and the global economy, but also caused global mental panic, especially for infected patients [2]. Active therapy is an effective mental health treatment method, which emphasizes the importance of people's natural potential in solving psychological problems. By stimulating people's cognitive ability and the ability of the object to love, they can reasonably and flexibly master and use methods such as environment, language, behavior, and drugs and take positive motivation or positive psychological suggestions to patients. Yin et al. believe that psychological intervention therapy based on the positive idea has been gradually introduced into various nursing fields at home and abroad and achieved good results in the research and practice progress of positive idea therapy in clinical medicine and nursing. It provides a reference for the research progress of positive therapy and its research and practice in clinical medicine and nursing [3]. In the case of novel coronavirus pneumonia, Chen Lin et al. analyzed the posttraumatic growth status, stress disorder, and social support of patients with novel coronavirus pneumonia. Psychological factors have significant effects on traumatic stress disorder (PTSD) and social support on the posttraumatic growth of patients with COVID-19. It has a positive effect on the follow-up psychotherapy of patients, which can enable patients to achieve positive growth when experiencing this epidemic event [4]. Patients with novel coronavirus pneumonia were also treated with psychological intervention. Li Fang and others (2020) also considered that targeted psychological intervention was aimed at promoting psychological rehabilitation of patients with new crown pneumonia. At the same time, effective psychological intervention measures should be taken for posttraumatic growth [5]. During the epidemic period, long-term closed management is easy to control people's inner uneasiness and anxiety, which is not conducive to the development of mental health. Liuaibing reported that COVID-19 mainly infect the respiratory tract, digestive tract, and contact. According to relevant studies, people will have sympathetic excitement in a short time in the face of emergencies, but it will develop into a traumatic stress disorder after more than 30 days. Therefore, coronary pneumonia can easily lead to traumatic stress disorder [6]. In the study of Zhang Kai according to the questionnaire survey on the public during the new crown period, there are significant differences in emotional and behavioral responses among respondents of different genders. The emotional and cognitive responses in areas with serious epidemics are higher than those in low-risk areas. And there is obvious alternative trauma [7]. A large number of people are affected by the epidemic, and it is difficult to concentrate on work and study, thus losing the basic trust between people. The disorder caused by novel coronavirus pneumonia affects not only the physical and psychological aspects of infected individuals but also the psychological behaviors of the related personnel. It also endangers the daily life and economic functions of families, social groups, and the masses. In patients with COVID-19, there is a phenomenon of severe depression, which will lead to inability to take care of themselves, accompanied by strong autistic psychology. Novel coronavirus pneumonia was used to analyze posttraumatic growth in patients with positive coronavirus pneumonia. In the face of public social epidemics, people instinctively experience nervous excitement in a short time. During this period, people will not enter into an emotional trauma reaction. After this process lasts for a period of time, it will lead to anxiety, irritability, and depression. Timely posttraumatic psychiatric investigation and intervention can provide targeted treatment and prevention in advance. The aim of this study was to explore the correlation between posttraumatic stress disorder (PTSD) and the incidence of anxiety, depression, and mental disorders in patients with new crown pneumonia.

The article "Correlation Analysis of Positive Therapy Based on High Content Image Analysis Technology on Posttraumatic Nerve Growth in Patients with COVID-19 in the Context of Intelligent Medical Treatment" was published in 2022. Journal: Contrast Media Mol Imaging.

## 2. PTSD Performance and Problem Design of Patients Diagnosed and Rescued

PTSD generally refers to posttraumatic stress disorder. Posttraumatic stress disorder (PTSD) refers to the delayed and persistent mental disorder caused by an individual's experience, encounter or witness of one or more actual deaths involving himself and others, or death threats, serious injuries, or threats to physical integrity. There are many factors for the occurrence of PTSD in severe patients. The main factors are family, social psychology, biological factors, etc. Among them, women are more likely to develop PTSD symptoms than men, and the major traumatic events experienced by patients are the basic condition for the onset of PTSD, which is seriously unpredictable [8]. In order to better treat and care patients, we observed the different performance of PTSD in the diagnosis of rescue patients, as shown in Table 1.

Table 1 shows the different manifestations of PTSD in patients diagnosed and rescued, such as the patient's response at the time of diagnosis and admission, observing whether the patient has no performance, anxiety, irritability, tremor, or syncope, and observing whether the patient has anxiety, irritability, tremor, and other manifestations when treating doctors, nursing nurses, and relevant environment and personnel.

The article "Correlation Analysis of Positive Therapy Based on High Content Image Analysis Technology on Posttraumatic Nerve Growth in Patients with COVID-19 in the Context of Intelligent Medical Treatment" was published in 2022. Journal: Contrast Media Mol Imaging.

## 3. PTSD Performance and Problem Design of Closely Connected and Isolated Patients

For novel coronavirus pneumonia patients with close isolation, better infection prevention and control will be the centralized management of suspected patients with close connection. The isolation points are generally designated by local governments with certain conditions for hotels, and close isolation observation is carried out to prevent the development and spread of the epidemic. Observe and analyze the different manifestations of PTSD of closely connected isolated patients at centralized closed isolation points, as shown in Table 2.

Table 2 shows the PTSD performance of close contact and isolated patients. The response of close contact patients to environmental sanitation at the isolation point during admission, closed management, management of relevant personnel, and the severity of anxiety, irritability, syncope, and other different manifestations of patients were observed in detail.

## 4. Performance and Problem Design of PTSD in Patients with Three Times Close Contact Isolation

People infected with new coronavirus have no symptoms during the incubation period, but they are infectious at this time. Therefore, patients in the incubation period become invisible virus communicators and are difficult to control. Ordinary personnel who have contacted such patients without protection become secondary close contacts. Family members and colleagues who have frequent contact with secondary close contacts are also the objects of secondary close contact isolation. All patients need to be isolated at home or observed in the community. The different observations of PTSD in patients with secondary close contact isolation are shown in Table 3.

Table 3 shows the different manifestations of PTSD in patients with secondary close contact isolation. Observe the response of patients with secondary close contact isolation, the response to community isolation personnel, the response to home closed isolation, the response of family members, and the response to environmental accommodation to find out the different manifestations of patients and the correlation degree of performance.

## 5. Scale Weighting Algorithm and Data Integration Method

The nursing staff observed the specific performance of the patient and checked it on the scale: no performance score: 0, anxiety score: 1, irritability score: 2, tremor score: 5, and syncope score: 10.

For 6 questions in each of the three groups of the above scale, the matrix structure is shown as follows:

(1) $$\begin{array}{c} M=\left\{\begin{array}{c} \left\{A_{i}=0,1,2,5,10\right\};i=1,2,3,4,5,6;\\ \left\{B_{i}=0,1,2,5,10\right\};i=1,2,3,4,5,6;\\ \left\{C_{i}=0,1,2,5,10\right\};i=1,2,3,4,5,6; \end{array}\right\}. \end{array}$$

*A*_*i*_ is the score of item I in group A; *B*_*i*_ is the score of item I in group B; *C*_*i*_ is the score of item I in group C.

The article "Correlation Analysis of Positive Therapy Based on High Content Image Analysis Technology on Posttraumatic Nerve Growth in Patients with COVID-19 in the Context of Intelligent Medical Treatment" was published in 2022. Journal: Contrast Media Mol Imaging.

Weighted fusion of the above matrix M, form the weighted results of the scale *J*_*A*_, *J*_*B*_, *J*_*C*_, and the weighting method is shown as follows:

(2) $$\begin{array}{c} \left\{\begin{array}{c} {\text{J}}_{\text{A}}=\sum_{\text{i}=1}^{6}\varphi_{\text{i}}{\text{A}}_{\text{i}},\sum_{\text{i}=1}^{6}\varphi_{\text{i}}=1\\ {\text{J}}_{\text{B}}=\sum_{i=1}^{6}\beta_{\text{i}}{\text{B}}_{\text{i}},\sum_{i=1}^{6}\beta_{\text{i}}=1\\ {\text{J}}_{\text{C}}=\sum_{i=1}^{6}\vartheta_{\text{i}}{\text{C}}_{\text{i}},\sum_{i=1}^{6}\vartheta_{\text{i}}=1 \end{array}\right... \end{array}$$

J_A_ is the weighted result of group A; J_B_ is the weighted result of group B; J_C_ is the weighted result of group C; *φ*_i_ is the weighted index of the *i* score in group A; *β*_i_ is the weighted index of the *i* score in group B; *ϑ*_i_ is the weighted index of the *i* score in group C.

The above content *J*_*A*_, *J*_*B*_, *J*_*C*_ perform secondary weighting calculation, as shown in the following formula:

(3) $$\begin{array}{c} \text{J}=\rho_{\text{A}}{\text{J}}_{\text{A}}+\rho_{\text{B}}{\text{J}}_{\text{B}}+\rho_{\text{C}}{\text{J}}_{\text{C}},\rho_{\text{A}}+\rho_{\text{B}}+\rho_{\text{C}}=1. \end{array}$$

*J* is the final weighting result and *ρ*_A_, *ρ*_B_, *ρ*_C_ are the secondary weighting coefficients of the weighting results of group A, group B, and group C, respectively;

## 6. Positive Therapy for Novel Coronavirus Pneumonia PTSD Treatment Path Design

The control group was treated with PTSD routine therapy, symptomatic psychological counseling treatment, antianxiety, and antidepression treatment, combined with a light and severe care path.

On the basis of the control group, the observation group introduced positive therapy and full perfusion therapy, that is, under the condition of deep hypnosis, the full perfusion method was used to increase the patient's tolerance to the fear-sensitive stimulation corresponding to PTSD, and active treatment with deep hypnosis can trigger high-intensity emotional response and consolidate the treatment effect through continuous training, so as to improve the patient's subjective control ability.

The biggest clinical risk of positive therapy is the risk of guiding and awakening intervention of deep hypnosis. Those who perform hypnosis should observe the patient's physical and mental state at any time and use EEG, ECG monitoring, and other auxiliary observations throughout the whole process. When it is found that the patient's anxiety and depression are strengthened, they should wake up in time and withdraw from hypnotic intervention. If necessary, symptomatic intervention drugs should be used to treat anxiety, depression, and neuroticism. After the patient wakes up, confirm the mental state of the patient, make an assessment, and supplement antianxiety and antidepression treatment if necessary.

The article "Correlation Analysis of Positive Therapy Based on High Content Image Analysis Technology on Posttraumatic Nerve Growth in Patients with COVID-19 in the Context of Intelligent Medical Treatment" was published in 2022. Journal: Contrast Media Mol Imaging.

The observation group determined the intervention frequency and time of hypnotherapy (including positive therapy and full perfusion therapy) according to the specific physical and mental states of the patients.

## 7. Evaluation Results and Clinical Verification of Scale

### 7.1. General Information of Patients

Novel coronavirus pneumonia patients in Wuhan were selected from 2020 to April. 70 rehabilitation patients from the hospital and isolation wards were selected as the subjects. They were randomly divided into 2 groups: the observation group and the control group. The average age of the 35 patients in the observation group was 31 + 3.4 years. All the patients were treated with positive therapy. The average age of 35 patients in the control group was 37 years (4.1 years). All the patients were treated by routine rehabilitation therapy. Patients with past mental history and other serious physical diseases were excluded. After obtaining their informed consent, the scale was evaluated intensively. The evaluation process was supervised by 5 doctors and 3 nurses trained uniformly.

Inclusion criteria were as follows: ① novel coronavirus pneumonia patients aged 18 years old were recruited; ② the patients who have clear consciousness and barrier-free communication; and ③ patients who signed informed consent and voluntarily participated in this study.

Exclusion criteria were as follows: ① patients in the treatment stage of other diseases and ② recent traumatic events (e.g., family accidents, natural and man-made disasters, etc.).

### 7.2. Evolution Law of Patients' Anxiety

Because the spread of novel coronavirus pneumonia is relatively subtle and the speed of transmission is very fast, it has caused panic to some extent. Especially, the patients diagnosed and closely connected are suffering from all kinds of mental pressure from society, family, and themselves. In the negative emotions of patients, anxiety also has a strong embodiment. The change law of patients' anxiety is shown in Table 4.

Novel coronavirus pneumonia patients' anxiety scale was visualized by objective analysis of the evolution of anxiety.  Figure 1 shows the visual comparison of SAS self-rating scale of patients.

The article "Correlation Analysis of Positive Therapy Based on High Content Image Analysis Technology on Posttraumatic Nerve Growth in Patients with COVID-19 in the Context of Intelligent Medical Treatment" was published in 2022. Journal: Contrast Media Mol Imaging.

Table 4 and Figure 1 show that most of the novel coronavirus pneumonia patients had a certain degree of anxiety. The anxiety of the two groups before and after treatment was not significantly different. After treatment, the treatment effect of the observation group was better than that of the control group. It shows that novel coronavirus pneumonia can reduce anxiety and the effect is obvious.

### 7.3. Comparison of SAS Distribution after Treatment

The depression of patients after treatment was observed and analyzed, and the specific performance of patients was observed by medical staff for evaluation and scoring. Those with scores <4 had mild anxiety, and there was no significant difference between them and normal people; those with scores between 4 and 7 had moderate anxiety, and those with scores >7 had severe anxiety. Intervention treatment is also needed. The distribution of SAS after treatment is shown in Table 5.

The SAS distribution comparison table of anxiety patients after treatment is visualized, and Figure 2 is obtained.

Table 5 and Figure 2 show the distribution and comparison of SAS after treatment. The number of patients in the observation group with score <4 is significantly lower than that in the control group, and the number of patients with severe anxiety with score >7 is less than that in the control group. It proves that the treatment effect is better after the introduction of positive therapy and full perfusion therapy, which reduces the degree of anxiety and improves the cure success rate of patients.

### 7.4. Evolution Law of Patients' Depression

During the 2019 coronavirus disease period, due to different risk areas, unstable work income, lack of freedom to go out, and other unstable factors, it will also bring serious psychological burden to patients. If patients cannot adjust themselves in time and take intervention measures, they may cause depression and may gradually aggravate their depression. Patients' SDS self-rating scale is compared in Table 6.

Novel coronavirus pneumonia patients with depression were compared with the SDS self-rating scale, and it is shown in Figure 3.

In Table 6 and Figure 3, the results showed that there was no significant difference in the depression performance between the two groups before treatment. After treatment, the depression results of the observation group were significantly lower than those of the reference group. It shows that positive therapy has an obvious intervention effect on patients' depression, reduces patients' depression, and promotes patients' mental recovery.

### 7.5. Incidence Regularity of Patients with Severe Psychosis

If the anxiety, irritability, depression, and other conditions of PTSD in patients with new crown cannot be effectively controlled, the latter mental disorder may develop into severe schizophrenia, major depression, secondary antisocial personality, personality split, and other severe psychosis, which will cause injury and death and panic to the society to a certain extent. The comparison of the incidence of severe psychosis in patients is shown in Table 7.

The article "Correlation Analysis of Positive Therapy Based on High Content Image Analysis Technology on Posttraumatic Nerve Growth in Patients with COVID-19 in the Context of Intelligent Medical Treatment" was published in 2022. Journal: Contrast Media Mol Imaging.

According to the visualization of the comparative data results of severe psychosis in patients with Xinguan, Figure 4 is obtained.

In Table 7 and Figure 4, the observation group showed that there was no difference in the PTSD performance before and after treatment, but the treatment effect of the observation group was significantly better than that of the control group. The observation group was beneficial to the treatment of the new crown after introducing positive therapy, and it could greatly reduce the incidence rate of severe mental illness and play a positive role in social stability.

## 8. Discussion on the Application Effect of Scale

Because novel coronavirus pneumonia is a new type of virus, its understanding is not comprehensive enough, and the treatment of new crown pneumonia is still in the exploratory stage. These external and internal factors have unwittingly increased people's fear of it and increased their psychological burden [9]. In particular, novel coronavirus pneumonia patients are more intense in various aspects of posttraumatic growth, such as anxiety, irritability, depression, and syncope, which have a serious impact on their physical and mental health. As the biggest victim of the epidemic, society and relevant medical staff need to strengthen psychological counseling for patients with new coronavirus pneumonia, guide and help patients improve disease prevention knowledge, make rational use of social resources, and help patients gain positive growth from the experience of the epidemic [10]. Novel coronavirus pneumonia should be given more psychological support during the postepidemic period (Li and others). Patients with anxiety, depression, and PTSD should be focused on. The medical staff should take measures to improve their perceived social support level to alleviate posttraumatic stress disorder [11]. In the study of Chen et al., the novel coronavirus pneumonia has a higher incidence of unhealthy mental state. It is the result of multiple factors. Clinical intervention should be directed against all risk factors to alleviate the patient's bad mood [12]. Through the psychological intervention and statistics of patients in advance, we can understand the psychological changes of patients and carry out targeted guidance and treatment. It is convenient for the early diagnosis and treatment of posttraumatic stress disorder caused by COVID-19. It not only improves the mental health level of patients, but also plays an enlightening role in the intervention of posttraumatic growth of the public.

The article "Correlation Analysis of Positive Therapy Based on High Content Image Analysis Technology on Posttraumatic Nerve Growth in Patients with COVID-19 in the Context of Intelligent Medical Treatment" was published in 2022. Journal: Contrast Media Mol Imaging.

## 9. Summary

Based on the novel coronavirus pneumonia patients' conventional treatment, the study introduced positive therapy and full irrigation therapy to enable patients to increase their tolerance to PTSD performance to be sensitive to fear, anxiety, depression, and other sensitive stimuli under deep hypnosis condition. At any time, the mental state and physical state of patients were observed to improve their subjective control. By evaluating and scoring the PTSD performance of different patients, and comparing the results of SAS self-rating anxiety scale, SAS posttreatment distribution, SDS self-rating depression scale, and patients with severe psychosis, it was found that the treatment effect of the active treatment observation group was significantly better than that of the conventional treatment control group. Active treatment can enhance the patients' mental self-regulation ability and help them overcome negative emotions such as anxiety, irritability, and depression and reduce the mental internal friction of patients. Active treatment of novel coronavirus pneumonia has a positive effect on the posttraumatic growth of patients with COVID-19 pneumonia, relieving anxiety and negative emotions, improving emotional control, eliminating negative emotions, actively guiding patients, and promoting their psychological rehabilitation.

## Figures and Tables

**Figure 1:** Visual comparison of SAS self-rating scale of patients.

**Figure 2:** Visual diagram of SAS distribution comparison table after treatment.

**Figure 3:** Visual comparison of patients' SDS self-rating scale.

**Figure 4:** Visual comparison of patients with severe psychosis.

**Table 1:** Observation of PTSD performance of patients diagnosed and rescued.

ID	Performance issues/observations	No performance	Anxious	Grumpy	Tremor	Syncope
A1	Response of confirmed patients to admission	□	□	□	□	□
A2	Reaction to doctor's treatment	□	□	□	□	□
A3	Response to nurse care	□	□	□	□	□
A4	Response to the hospital environment	□	□	□	□	□
A5	Response to the ward and patient clothing	□	□	□	□	□
A6	Response to other hospital personnel	□	□	□	□	□

**Table 2:** Observation table of PTSD performance of closely connected and isolated patients.

ID	Performance issues/observations	No performance	Anxious	Grumpy	Tremor	Syncope
B1	Response of close contact patients at admission	□	□	□	□	□
B2	Response to the hotel, hotel environment, and sanitation	□	□	□	□	□
B3	Response to hotels and hotel service personnel	□	□	□	□	□
B4	Response to closed management	□	□	□	□	□
B5	Response to isolation management	□	□	□	□	□
B6	Response to accommodation at the isolation point	□	□	□	□	□

The article "Correlation Analysis of Positive Therapy Based on High Content Image Analysis Technology on Posttraumatic Nerve Growth in Patients with COVID-19 in the Context of Intelligent Medical Treatment" was published in 2022. Journal: Contrast Media Mol Imaging.

**Table 3:** Observation table of PTSD performance of patients with close contact isolation.

ID	Performance issues/observations	No performance	Anxious	Grumpy	Tremor	Syncope
C1	Response of patients with secondary close contact during isolation	□	□	□	□	□
C2	Response to community isolation	□	□	□	□	□
C3	Response to community isolation	□	□	□	□	□
C4	Response to isolated enclosed spaces at home	□	□	□	□	□
C5	Reaction to family in isolation	□	□	□	□	□
C6	Response to accommodation during isolation	□	□	□	□	□

**Table 4:** Comparison of SAS self-rating scale of patients.

Group	*n*	Before treatment	After treatment
Observation group	35	7.25 ± 0.92	4.33 ± 0.54
Control group	35	7.37 ± 0.87	5.28 ± 0.63
t value		25.364	5.243
*P* value		0.013	0.007

**Table 5:** Comparison of SAS distribution after treatment.

Group	*n*	SAS distribution after treatment		
		<4	4–7	>7
Observation group	35	27(77.1)	7(20.0)	1(2.85)
Control group	35	21(60.0)	9(25.7)	5(14.2)
t value		7.124	6.784	7.465
*P* value		0.006	0.007	0.008

**Table 6:** Comparison of SDS self-rating scale of patients.

Group	*n*	Before treatment	After treatment
Observation group	35	7.14 ± 0.86	4.58 ± 0.65
Control group	35	6.97 ± 0.93	5.34 ± 0.71
*t* value		21.045	6.382
*P* value		0.007	0.008

**Table 7:** Comparison of patients with severe psychosis.

Group	*n*	Before treatment	After treatment
Observation group	35	6(17.1)	1(2.9)
Control group	35	6(17.1)	3(8.6)
*t* value		7.168	6.472
*P* value		0.008	0.009

## Data Availability

The data underlying the results presented in the study are available within the manuscript.
